The article "Modulation of the Default Mode Network in First-Episode, Drug-Naïve Major Depressive Disorder via Acupuncture at Baihui (GV20) Acupoint" was published in 2016. Journal: Front Hum Neurosci.

# Modulation of the Default Mode Network in First-Episode, Drug-Naïve Major Depressive Disorder via Acupuncture at Baihui (GV20) Acupoint

**DOI:** 10.3389/fnhum.2016.00230

**Published:** 2016-05-17

**Authors:** Demao Deng, Hai Liao, Gaoxiong Duan, Yanfei Liu, Qianchao He, Huimei Liu, Lijun Tang, Yong Pang, Jien Tao

**Affiliations:** ^1^Department of Radiology, First Affiliated Hospital, Guangxi University of Chinese MedicineNanning, China; ^2^Life Science Research Center, School of Life Science and Technology, Xidian UniversityXi’an, China; ^3^Department of Internal Neurology, First Affiliated Hospital, Guangxi University of Chinese MedicineNanning, China; ^4^Department of Acupuncture, First Affiliated Hospital, Guangxi University of Chinese MedicineNanning, China

**Keywords:** acupuncture, Baihui, fMRI, functional connectivity, major depressive disorder

## Abstract

**Background**: Previous neuroimaging studies have revealed that acupuncture modulates the default mode network (DMN) in healthy subjects and patients with certain disorder. However, few studies have been performed to investigate whether or not acupuncture might modulate the DMN in patients with major depressive disorder (MDD). Thereby, the aim of the present study was to assess alterations of the DMN induced by acupuncture stimulation in patients with first-episode, drug-naïve MDD.

**Materials and Methods**: Twenty nine patients with first-episode, drug-naïve MDD and 29 healthy subjects were enrolled in this study. All the healthy subjects underwent 6-min resting-state functional magnetic resonance imaging (R-fMRI) scan. While patients underwent acupuncture stimulation for 20-min electro-acupuncture stimulation (EAS) at Baihui acupoint (GV20) and two 6-min R-fMRI scans before and after EAS. Based on the precuneus/posterior cingulate cortex (PC/PCC) as the seed region, functional connectivity (FC) method was adopted to examine abnormal DMN in patients by comparing with healthy subjects and to evaluate the influence of EAS on intrinsic connectivity within the DMN in patients with MDD.

**Results**: Compared to healthy subjects, MDD patients had abnormal DMN. Moreover, results showed that EAS at GV20 induced increased FC between the PC/PCC and bilateral anterior cingulate cortex (ACC), and decreased FC between the PC/PCC and left middle prefrontal cortex, left angualr gyrus and bilateral hippocampus/parahippocampus (HIPP/paraHIPP) in patients with MDD, which were the main brain regions showing significant differences between the patients and healthy subjects.

**Conclusion**: Our findings provide imaging evidence to support that GV20-related acupuncture stimulation may modulate the DMN in patients with first-episode, drug-naïve MDD. This study may partly interpret the neural mechanisms of acupuncture at GV20 which is used to treat patients with MDD in clinical.

## Introduction

As a debilitating psychiatric disorder, major depressive disorder (MDD) is characterized by depressed mood, anhedonia, irritability, difficulties in concentration, and abnormalities in appetite and sleep (Nestler et al., 2002). MDD has a negative effect on the quality life of patients and leads to a huge economic burden for patient’s family (Collins et al., 2011). MDD will become the second cause of burden of disease by 2030 (Mathers and Loncar, 2006). Recent large-scale epidemiological surveys in China have shown that the prevalence of MDD patients is high to 6.1%, which causes many social problems (Phillips et al., 2009). Thus, it is necessary to pay more attention to understanding the pathophysiological mechanisms of MDD and finding effectively therapeutic approaches.

As one of the most commonly recognized resting-state networks, the default mode network (DMN) comprises the brain areas mainly including the middle prefrontal cortex, anterior cingulate cortex (ACC), posterior cingulate cortex (PCC), precuneus (PC), angular gyrus and inferior parietal cortex (IPC; Raichle et al., 2001; Greicius et al., 2003). The DMN plays an important role in self-referential activities, such as evaluating characteristics of external and internal cues, planning the future, and remembering the past (Raichle and Snyder, 2007; Buckner et al., 2008). Recently, several studies have revealed dysfunctional DMN in MDD patients, and altered functional connectivity (FC) between brain regions were mainly located in the middle prefrontal cortex, angular gyrus, ACC and hippocampus (HIPP; Anand et al., 2005a; Tahmasian et al., 2013; Jacobs et al., 2014; Khalsa et al., 2014; Chen et al., 2015; Sankar et al., 2015). The aforementioned studies indicated that the DMN was one of the most mature network matched with functional magnetic resonance imaging (fMRI) for studying mechanisms of MDD (Guo et al., 2014; Chen et al., 2015) and suggested that abnormal DMN was associated with MDD.

As one complementary and alternative therapy method, acupuncture may improve microcirculation, balance organ function, and adjust mental activities. Acupuncture thereby has been increasingly and widely accepted by western countries (Lee et al., 2014). Neuroimaging technologies have been used to investigating neural mechanisms of acupuncture, and it has been found that acupuncture stimulation may modulate the DMN in healthy subjects and patients with certain psychiatric disorders, such as stroke, migraine and Alzheimer’s disease (AD; Dhond et al., 2008; Fang et al., 2009; Hui et al., 2009; Liu et al., 2009b; Wang et al., 2014; Zhang et al., 2014).

According to traditional Chinese medicine theory, Baihui acupoint (GV20) is located at the highest place of the head, and GV20 is a commonly acupoint used to relief of dizziness, headache and anxiety by acupuncture stimulation, which attributes to the effect of acupuncture at GV20 on modulating vascular, endocrine, immune and/or nervous systems (Satoh, 2009). GV20 was indentified to be involved in the treatment of MDD (Sun et al., 2013; Li et al., 2014). This raised the questions: whether or not the DMN could be modulated by acupuncture stimulation at GV20 in MDD patients. If so, how acupuncture stimulation modulated intrinsic connectivity in the DMN. To our knowledge, limited neuroimaging studies focused on relationships between the acupuncture stimulation at GV20 and the DMN in MDD patients.

In the present study, we tried to investigate whether or not acupuncture stimulation at GV20 could modulate the DMN in patients with first-episode, drug-naïve MDD using FC method. FC is known to describe relationships between the neuronal activation patterns of anatomically separated brain regions, showing the level of functional communication among regions (Van Den Heuvel and Pol, 2010). FC is typically used in most resting-state fMRI studies and is suitable for exploring the DMN (Greicius et al., 2003; Liu et al., 2009b; Van Den Heuvel and Pol, 2010; Sripada et al., 2014; Lehmann et al., 2015). Here, we hypothesized that the abnormal DMN in patients might be modulated by acupuncture, which might attribute to the characteristic of GV20.

## Materials and Methods

### Ethics Statement

All participants were informed about the whole experiment procedure and signed an informed consent. The current study was permitted by the Medicine Ethics Committee of First Affiliated Hospital, Guangxi University of Chinese Medicine, Guangxi, China. All research procedures of the current study were conducted in accordance with the Declaration of Helsinki.

### Subjects

Thirty patients with first-episode, drug-naïve MDD (21 females and 9 males) were recruited from out-patients or in-patients at Department of Internal Neurology, First Affiliated Hospital, Guangxi University of Chinese Medicine, Guangxi, China. All the patients were individually diagnosed by two trained psychiatrists using the structured clinical interview of the diagnostic and statistical manual of mental disorders-fourth criteria (DSM-IV; First MB et al., 1997). And the inclusion criterion for patients were: (1) being first-episode, drug-naïve; (2) the ages between 18 and 45 years; (3) being right-handed; and (4) having episode experience of MDD with the score of at least 18 on 17-items Hamilton Depression Rating Scale (HDRS-17; Guo et al., 2014). The exclusion criterion for patients were: (1) having other disorders by DSM-IV criteria, such as schizoaffective disorder, schizophrenia, organic mental disorder , delusional mental disorder, psychotic features coordinated or uncoordinated with mood or bipolar disorder; (2) having history of head injury or neurological disorder and degenerative diseases, such as movement disorder and Parkinson’s disease; (3) having acutely suicidal or homicidal tendency; (4) having any MRI contraindications; (5) having acupuncture contraindications; and (6) being non-responders in acupuncture needling.

Twenty nine healthy subjects (14 females and 15 males; mean age: 26.76 ± 1.72 years) were recruited in this study. All the healthy subjects were free of depression or other psychiatric or neurological illness, and had no history of head injury and alcohol or drugs abuse. Healthy subjects did not have any family history related to neurological or psychiatric illness in their first-degree relatives.

In addition, it was required that all of the subjects were no smokers, current pregnancy or breast feeding. Meanwhile, each subject completed an identical assessment protocol, which including the HDRS-17, self-rating depression scale (SDS) and self rating anxiety scale (SAS; Guo et al., 2013b).

### Experiment Paradigm

Each healthy subject underwent only a 6-min resting-state scan. While each patient underwent two 6-min resting-state scans before and after the acupuncture stimulation for 20-min electro-acupuncture stimulation (EAS) at GV20. In detail, this study focused on GV20, which was a point on the Governor Vessel and located on the vertex of the head (Satoh, 2009; Figure 1A). The non-repeated event-related (NRER) paradigm was applied in the study (Qin et al., 2008; Liu et al., 2009a). Twenty minutes (20-min) EAS at GV20 was operated by the same professional acupuncturist (1 Hz, 2 mA, continuous-wave, HuaTuo-brand, SDZ-V-type, Shanghai, China; Figure 1B). EAS was performed by inserting the sterile stainless steel disposable needle (0.30 mm in diameter and 25 mm in length; Huatuo-brand, Suzhou, Jiangsu, China) into GV 20 at the depth of needling arranging from 1.0 cm to 1.5 cm. Another electrode was attached to the acupuncture needle which was shallowly inserted point 1.0 cm nearby GV20. During scanning, each patient was instructed to keep eyes closed, not to think about anything and to stay awake. At the end of scanning, each patient was required to recall acupuncture sensations as following: aching, soreness, numbness, fullness, sharp or dull pain, pressure, heaviness, warmth, coolness, tingling, itching, and any others. The intensity of each sensation was measured by using a 100-point visual analog scale (VAS; 0 = no sensation, 10–30 = mild, 40–60 = moderate, 70–80 = strong, 90 = severe and 100 = unbearable sensation), which was similarly determined by Hui et al. (2005, 2007).

**Figure 1:** **(A)** Location of Baihui acupoint (GV20); **(B)** Experimental paradigm.

### MRI Data Acquisition

Images were acquired using a 3.0 Tesla Siemens Magnetom Verio MRI System (Siemens Medical, Erlangen, Germany) at the Department of Radiology, First Affiliated Hospital, Guangxi University of Chinese Medicine, Nanning, Guangxi, China. To reduce head movement, each subject’s head was fixed by foam pads in a standard 8-channel birdcage head coil. Functional images were acquired with a single-shot gradient–recalled echo planar imaging (EPI) sequence with the parameters: repetition time (TR)/echo time (TE) = 2000/30 ms, Flip angle = 90°, field of view (FOV) = 240 mm×240 mm, matrix size = 64 × 64, slice thickness = 1 mm and slices = 31. High resolution T1-weighted images were then collected with a volumetric three-dimensional spoiled gradient recall sequence with the parameters: TR/TE = 1900/2.22ms, FOV = 250 mm×250 mm, matrix size: 250 × 250, flip angle = 9°, slice thickness = 1 mm and 176 slices).

### Image Preprocessing

Statistical parametric mapping software (SPM8)^1^ and REST toolbox (REST 1.7)^2^ were used to analyze functional images. The first 10 functional volumes were removed for stabilization of the initial signal. Then the remaining volumes were corrected by slice timing and then realigned to correct for head motion. Data with maximum displacement in any directions of larger than 2 mm or head rotation of larger than 2° were excluded from further analysis. The datasets were further spatially normalized to the Montreal Neurological Institute (MNI) template and resampled to 3 × 3 × 3 mm^3^ isotropic voxels. The normalized data were smoothed with a 4-mm full width at half maximum (FWHM) Gaussian kernel. Nuisance covariates were regressed out from our data, including the six head motion parameters, white matter signal and cerebrospinal fluid (CSF) signal. As global signal regression may cause a negative shift in the distribution of correlations (Murphy et al., 2009; Saad et al., 2012, 2013), global signal was not regressed in our study. The data were then detrended and bandpass filtered from 0.01 to 0.08 Hz to reduce the effect of low-frequency drifts and high-frequency noise.

### Functional Connectivity Analysis

To identify the DMN, the seed region was selected in the PC/PCC (Sheline et al., 2010). The mean blood-oxygen-level dependent (BOLD) time course was extracted from a 6 mm sphere in the selected PC/PCC (MNI coordinates: −9, −60, 25) of each subject on different conditions, including one resting-state condition in healthy subjects and two resting-state conditions before and after EAS in patients. Pearson correlation coefficients were estimated between the mean time course of the seed region and the time course of all the other voxels within the whole brain based on different subjects and conditions, separately. Pearson correlation coefficients were then normalized to *z*-scores with Fisher’s *r*-to-*z* transformation to acquire the entire brain *z*-score map of each subject on each condition.

### Statistical Analysis

Demographic and clinical data were compared by using two-sample *t*-test and Chi-square test. The threshold level in all statistical analysis for significance criterion was determined at *p* < 0.05. Main acupuncture sensations were described with each sensation intensity and frequency in patients.

To explore the DMN, one sample *t*-test was firstly used for FC maps from healthy subjects, patients and patients after EAS, respectively. Two sample *t*-test was then applied to examine different patterns of the DMN between patients and healthy subjects. Paired *t*-test was used to examine the modulated patterns of the DMN in patients before and after EAS. The contrast map was thresholded at a voxel-level threshold of 0.005 with a cluster-level threshold of 0.05 (false discovery rate (FDR) corrected). The age, gender, weight, SAS and SDS were deemed as covariates of no interest.

## Results

### Demographic and Clinical Results

In our study, one patient was excluded from further data analysis because of incomplete EAS at GV20 during the experiment. There were no significant differences in terms of age, gender and weight between the patients and healthy subjects. Patients had higher scores in HDRS-17, SDS and SAS compared to healthy subjects (Table 1).

**Table 1:** **Demographic and clinical characteristics for the study**.

Variable	HSs (*n* = 29)	DPs (*n* = 29)	*p* value
Gender (male/female)	15/14	9/20	0.182^a^
Age (years)	26.76 ± 1.72	28.69 ± 6.69	0.138^b^
Weight (kg)	59.55 ± 12.95	55.10 ± 10.50	0.157^b^
SDS	42.17 ± 7.74	62.72 ± 9.81	<0.001^b^
SAS	43.00 ± 7.59	62.14 ± 8.79	<0.001^b^
HDRS-17	4.48 ± 3.22	21.31 ± 2.58	<0.001^b^

*Abbreviations: SDS, self rating depression Scale; SAS, self rating anxiety scale; HDRS, hamilton depression rating scale; HSs, healthy subjects; DPs, major depressive disorder patients. Except for gender, all values are mean ± standard deviation (SD). ^a^The p-value was obtained by Chi-square. ^b^The p-value was obtained by two sample t-test*.

### Acupuncture Sensations Results

The prevalence of *Deqi* sensations reported by patients was expressed as frequency and intensity (Figure 2). The current results showed that main *Deqi* sensations included fullness, dull pain, numbness, soreness, tingling and heaviness.

**Figure 2:** **Results of acupuncture sensations in patients with major depressive disorder (MDD).** The soreness, numbness, fullness and dull pain were primary *Deqi* sensations. **(A)** The frequency of acupuncture sensations in patients with MDD. **(B)** The intensity of acupuncture sensations in patients with MDD.

### Imaging Results

The patterns of the DMN in both healthy subjects and patients are shown in Figure 3. The DMN mainly consisted of the middle prefrontal cortex, ACC, medial temporal cortex (MTC), bilateral angular gyrus. Compared to healthy subjects, patients had significantly statistical increased FC between the PC/PCC and the right middle prefrontal cortex and bilateral angular gyrus, and decreased FC between the PC/PCC and bilateral ACC (Figure 4A and Table 2). When it came to acupuncture stimulation, EAS-related results showed decreased FC in the left middle prefrontal cortex, left angular gyrus and bilateral HIPP/paraHIPP with the PC/PCC, and increased FC in the bilateral ACC with the PC/PCC in patients (Figure 4B and Table 2).

**Figure 3:** **The default mode network (DMN). (A)** The DMN in healthy subjects; **(B)** the DMN in patients with first-episode, drug-naïve MDD; **(C)** the DMN in patients with first-episode, drug-naïve MDD after electro-acupuncture stimulation (EAS) at Baihui (GV20).

**Figure 4:** **Distinct brain regions. (A)** Differences of the DMN between patients and healthy subjects; **(B)** differences of the DMN in patients before and after EAS at Baihui (GV20).

**Table 2:** **Main localization of default mode network (DMN) maps by comparing patients with healthy subjects and comparing electro-acupuncture stimulation (EAS) with resting state in patients**.

			MNI		
Regions	Hem	BA	*X*	*Y*	*Z*	*T*-Value	Vol
**Patients vs. healthy subjects**
Middle prefrontal cortex	R	8	24	18	54	3.97	62
Angular gyrus	L	3/79	−36	−63	45	3.76	39
	R	39/7	42	−69	48	4.18	44
ACC	L	24/32	−6	36	12	−3.66	65
	R	24/32	6	42	6	−3.98	59
**EAS vs. resting in patients**
Middle prefrontal cortex	L	8	−21	18	51	−3.96	57
Angular gyrus	L	39/7	−39	−60	48	−4.78	92
ACC	L	24/32	−6	36	12	3.75	39
	R	24/32	6	33	21	4.1	46
HIPP/paraHIPP	L	36	−27	−18	−18	−3.96	38
	R	36	27	−15	−18	−3.82	33

*Abbreviation: Hem, hemisphere; BA, Brodmann area; Vol, voxels; ACC, anterior cingulate cortex; HIPP/paraHIPP, hippocampus/parahippocampus; EAS, electro-acupuncture stimulation*.

## Discussion

In line with the NRER-fMRI design paradigm, we investigated modulatory effect of EAS at GV20 on the intrinsic connectivity within the DMN in patients with first-episode drug-naïve MDD. We found: (1) compared to healthy subjects, patients had abnormal patterns of the DMN including the right middle prefrontal cortex, bilateral angular gyrus and ACC with the PC/PCC; (2) EAS at GV20 modulated the DMN in patients, related to the left middle prefrontal cortex, left angular gyrus, bilateral HIPP/paraHIPP and ACC. Our findings provided further imaging evidence to support the neural mechanisms of GV20 on modulating abnormal DMN in MDD patients.

### Abnormal DMN in Patients

Compared to healthy subjects, MDD patients had abnormally increased/decreased FC regions associated with the middle prefrontal cortex, angular gyrus and ACC in this study. Previous studies had found altered DMN in patient with depression (Greicius et al., 2007; Bluhm et al., 2009; Sheline et al., 2010; Zhou et al., 2010). Our findings were similar to the results from these previous studies. Prefrontal cortex is involved in integration of cognitive, emotional behaviors by uniting emotional biasing signals or markers into decision making processing (Gusnard et al., 2001; Simpson et al., 2001). As one important part of IPC, angular gyrus plays a critical role in biological substrates of language, thought, attention and spatial working memory (Niznikiewicz et al., 2000), and is also enrolled in many diverse different tasks, such as the perception of emotions and interpretation of sensory information (Müller et al., 2013; Passingham et al., 2014; Ruschel et al., 2014). Recently, dysregulation of the IPC was found in depression and schizophrenia (Müller et al., 2013). Angular gyrus exhibited a more abnormal FC in depression patients (Guo et al., 2013a), and the parietal cortex systems showed hyperconnectivity with regions of the DMN in MDD patients (Kaiser et al., 2015). Thereby, increased FC of the prefrontal cortex and angular gyrus in our study might suggest that MDD patients could have dysfunctions of cognitive and emotional system. Meanwhile, our results showed significantly decreased FC in the ACC with the PC/PCC in patients. ACC is known to be one of the most important regions related to cognition, emotion and memory (Davis et al., 2005; Greicius et al., 2007; Lavin et al., 2013). Decreased connectivity of ACC with limbic regions was also found in patients with depression (Anand et al., 2005b). Thereby, we further speculate that decreased FC in the ACC is likely involved in the pathological mechanisms of MDD.

### Modulation on the DMN in Patients after EAS

After 20-min EAS, the DMN patterns in patients were modulated. Results showed that the significantly decreased FC between the PC/PCC and the left middle prefrontal cortex, left angular gyrus and bilateral HIPP/paraHIPP in MDD patients after EAS at GV20. The present findings were similar to the ones from several previous studies, which reported that acupuncture stimulation induced signal attenuation in the middle prefrontal cortex, HIPP/paraHIPP and IPC (Wu et al., 1999; Yoo et al., 2004; Hui et al., 2009). HIPP/paraHIPP is implicated in cognitive-behavioral functions and emotional memory (LaBar and Cabeza, 2006; Savitz and Drevets, 2009). Impaired function of the HIPP/paraHIPP was found in MDD patients (Hamilton and Gotlib, 2008). On the other hand, positive artificial intervention improved status for MDD patients due to excellent performance of angular gyrus (Shen et al., 2015). Therefore, the decreased FC between the PC/PCC and middle prefrontal cortex, angular gyrus and HIPP/paraHIPP in our study might indicate the positive effect of GV20-related acupuncture on eliminating formatted negative emotion and mediating memory related to depression. Our findings also showed that there were significantly increased FC in the ACC with the PC/PCC in patients after EAS. It had been reported that increased FC was found in ACC within the DMN in depression patients after artificial intervention, such as task stimulation and antidepressant treatment (Anand et al., 2007; Greicius et al., 2007; Zeng et al., 2012). Our findings could present that there might exist positive intervention effects on the ACC of MDD patients, which were attributed to acupuncture at GV20.

There were some limitations of our study: (1) Our study aimed to investigate whether or not GV20-related acupuncture stimulation might modulate the DMN in MDD patients, but not to investigate the specificity of acupoint (GV20). So, there was not a sham acupoint as a control in our experiment paradigm. However, the acupuncture associated with both GV20 and sham acupoint was our another research target in the future; (2) There were not different gender distributions of the two groups. Although gender, as a nuisance covariate, was regressed out from our data, gender factor could still not fully eliminate. Gender differences should be investigated and the present findings should be retested in larger samples in the future; and (3) The present results showed a preliminary research about the immediate effect of EAS on the DMN in patients with MDD. Further studies were still needed to confirm whether or not there were the possibilities of improving treatment effect in patients by a long-term EAS at GV20.

## Conclusion

We used fMRI and FC method to investigate the modulation mechanisms of GV20-related EAS to the DMN in MDD patients. Results showed EAS induced altered FC in the DMN, including the middle prefrontal cortex, angular gyrus, ACC and HIPP/paraHIPP which were the main regions showing abnormalities between patients and healthy subjects. Our findings might provide imaging evidence to support that EAS at GV20 has intervention effect on the DMN in patients with first-episode, drug-naïve MDD.

## Author Contributions

DD made substantial contributions to the overall conception of the work, designed the experiment, revised and handled the manuscript, accurately answered all the questions from the reviewers, ensured the integrity of the work, and approved the final version to be published. HL made important contribution to the literature review, interpreted data for the work, drafted the manuscript, revised some critical structure and intellectual content, advised on the integrity of the work, and approved the final version to be published. GD made important contribution to the design of MR scan protocols, carried out MRI operation, MRI data acquisition and storage, and approved the final version to be published. YL conducted the data processing and analysis for the functional MRI data, interpreted the conceptions of data processing, wrote the procedure of data processing, and approved the final version to be published. QH executed the diagnosis of patients, recruited subjects for this study, interpreted intellectual content in depression, was accountable for some aspects of the work in ensuring that questions related to the accuracy of the work were appropriately resolved, and approved the final version to be published. YP provided the acupuncture theory, made substantial contributions to the overall design and guideline of acupuncture experiment, interpreted intellectual content in acupuncture, and approved the final version to be published. HL was responsible for acupuncture operations, advised on the improvement of acupuncture protocols, provided important intellectual content in acupuncture, and approved the final version to be published. LT and JT conducted the assessment of acupuncture sensations, gave some important advice for the accuracy interpretation or description of conceptions related to acupuncture theory, and approved the final version to be published.

## Conflict of Interest Statement

The authors declare that the research was conducted in the absence of any commercial or financial relationships that could be construed as a potential conflict of interest.

## Footnotes

^1^http://www.fil.ion.ucl.ac.uk/spm

^2^http://www.resting-fmri.sourceforge.net

## Abbreviations

ACC: Anterior cingulate cortex
DMN: Default mode network
EAS: Electro-acupuncture stimulation
FC: Functional connectivity
HDRS-17: 17-items Hamilton Depression Rating Scale
HIPP/paraHIPP: Hippocampus/parahippocampus
MDD: Major depressive disorder
PC/PCC: Precuneus/posterior cingulate cortex
R-fMRI: Resting-state functional magnetic resonance imaging
SAS: Self rating anxiety scale
SDS: Self-Rating Depression Scale.
